The article "Purification and Analysis of the CREPT Antibody from Mouse Ascites" was retracted in 2023. Reasons: signs of a paper mill; suspected computer-generated content; unreliable results or conclusions; concerns about the data.

# Purification and Analysis of the CREPT Antibody from Mouse Ascites

**DOI:** 10.1155/2022/8776565

**Published:** 2022-09-05

**Authors:** Zhihao Xie, Jun Li, Xinbao Hao, Lu Xu

**Affiliations:** ^1^Department of Hematology, The First Affiliated Hospital of Hainan Medical University, Haikou 570102, Hainan, China; ^2^State Key Laboratory of Membrane Biology, School of Medicine, Tsinghua University, Beijing 100091, China

## Abstract

**Methods:**

Cells were cultivated properly to obtain 3E10 CREPT monoclonal antibody cells in the logarithmic growth stage. Monoclonal antibody cells were injected into the abdominal cavity of sensitized mice. The flowing ascites were observed for 7-15 days. The antibody protein was obtained by collection, filtration, dilution, loading, and chromatography. Furthermore, its binding force was detected by SDS-PAGE and Western blot techniques.

**Results:**

The antibody protein was successfully obtained with a purity of 1895 *μ*g/mL with high liveness.

**Conclusion:**

This study establishes a one-step purification method for obtaining monoclonal antibody with high liveness and purity for CREPT ascites antibody. This method is simple to perform and lays a foundation for the preparation and purification of humanized monoclonal antibodies in the future. In addition, it provides a basis for further research to investigate how CREPT affects the occurrence and development of different tumors.

## 1. Introduction

Cell-cycle related and expression-elevated protein in tumor (CREPT), also known as RPRD1B, is a newly discovered gene closely related to tumors in recent years [1]. The size of the CREPT gene is about 978 bp, and it encodes a protein of about 37 KB with a sequence of 326 amino acids. CREPT is found in many tumor tissues and is a protooncogene involved in the cell cycle [2]. Through genetic analysis, CREPT, p15RS, and RTT103 evolved in the same progenitor cells and participated in cell cycle regulation. Previous studies have found that CREPT is involved in various regulations of transcription, cell cycle, tumorigenesis, and DNA repair [3, 4]. CREPT is a cell cycle-related protein. The occurrence and development of tumors are closely related to the cell cycle. The formation of tumors is a multifactor, multistage, and multigene process. During the cell cycle, oncogenes and tumor suppressor genes are regulated [5, 6].

Accompanied by the activation of oncogenes, the inactivation of tumor suppressor genes, and the disorder of the cell cycle, CREPT is one of the proteins involved in the regulation of the cell cycle. Through previous studies, it was found that the overexpressed CREPT gene can accelerate the cell cycle and promote the occurrence and development of tumors. Preliminary laboratory ChIP experiments have shown that CREPT binds to the promoter of cyclin (cyclin D1) during the cell cycle and accelerates its transcription, thereby increasing the expression level of cyclin D1 and participating in the regulation of tumor occurrence and development [7]. To the best of our knowledge, there has been no reports on the purification and analysis of CREPT antibodies from mice ascites. This study is aimed at establishing a method for purification of CREPT antibodies from mouse ascites. Ascites were induced in mice with the CREPT monoclonal antibody cells produced in the laboratory, the antibody protein was also collected, separated, and purified, and the antibody protein was obtained, identified, and analyzed, which provided the experimental basis for the next research.

The article "Purification and Analysis of the CREPT Antibody from Mouse Ascites" was retracted in 2023. Reasons: signs of a paper mill; suspected computer-generated content; unreliable results or conclusions; concerns about the data.

## 2. Materials and Methods

### 2.1. Laboratory Reagents and Equipment

CREPT monoclonal antibody cells (3E10) from the monoclonal antibody cell line were obtained from Professor Chang Zhijie's laboratory at Tsinghua University. Other reagents including MOLT-4 (human acute lymphoblastic leukemia cells), 1640 medium, penicillin-streptomycin, and fetal bovine serum (FBS) were obtained from Grand Island Biological Company through local supplier. Incomplete Freund's adjuvant was acquired from Sigma, RPRD1B antibody from Invitrogen, horseradish peroxidase-labeled goat anti-mouse IgG (H + L) and RIPA lysis solution from Biyuntian, physiological saline from Biyuntian, NAb™ Spin Kits, 1 mL for antibody purification from Thermo Fishery, and BALB/c-nu from Hunan Slike Jingda Laboratory Animal Co., Ltd.

Ultraclean workbench (Thermo Fisher); desktop high-speed refrigerated centrifuge (5430R Eppendorf); cell inverted microscope (IX73 + DP22 Olympus); medical cryogenic refrigerator (Thermo Fisher); CO_2_ incubator (Thermo Fisher); liquid nitrogen tank (Thermo Fisher); inverted fluorescence microscope (Axio Observer3 Zeiss); ultrasonic disruptor (VCX130 US SONICS); full wavelength microplate reader (Varioskan LUX Thermo Fisher Scientific); multifunctional gel imager (AI680RGB GE); Mini-PROTEAN, Tetra System Protein Electrophoresis Instrument, and Trans-Blot TurboTM Protein Transfer Instrument (Bole Life Medical Products Co., Ltd.); water bath (Shanghai Boxun); mouse IVC (Suhang); and vertical pressure steam sterilizer (MVS83 Panasonic Cold Chain) instruments were used in this research.

### 2.2. Cell Culture

Cell culture medium was 10% FBS and 90% 1640 basal medium. CREPT mAb cells (3E10) were removed from liquid nitrogen and placed in a 37°C water bath to rapidly lyse the cells. After the cells were completely lysed, they were transferred to a sterile ultraclean bench and transferred to a 15 mL centrifuge tube in a sterile environment. Serum-containing medium was added, mixed well, and centrifuged at 1000 rpm/min for 5 minutes. Cells were suspended in a 1640 medium containing 10% FBS and collected by centrifugation. 10% FBS 1640 medium was added and cultured in a saturated humidity incubator at 37°C in a 5% CO_2_ atmosphere. The medium was changed every 2-3 days, and the cells were observed. Cells were passaged in the logarithmic growth phase, and the cells in the logarithmic growth phase were taken as the experimental research objects.

The article "Purification and Analysis of the CREPT Antibody from Mouse Ascites" was retracted in 2023. Reasons: signs of a paper mill; suspected computer-generated content; unreliable results or conclusions; concerns about the data.

### 2.3. Preparation of Mouse Ascites

BALB/c female mice (*n* = 3; 6-8 weeks old) were selected, and they were intraperitoneally injected with Freund's incomplete adjuvant (Sigma) at 0.5 mL/mice dose and injected hybridoma cells for around 7-20 days. The hybridoma cells in the logarithmic growth phase were taken, washed with normal saline, and adjusted to a cell concentration of 10^6^ cells/mL. Each mouse was injected with 1 mL, for a total of 3 mice. During this period, the activity and feed intake of the mice were observed [8, 9]. After 7-15 days of injection of cells in mice, the abdomen was bulging, and there were obvious mobile ascites. During this period, ascites can be placed 2-3 times, about 2 mL each time. The ascites were centrifuged (2000 rpm/min, 5 min) to remove cellular components and other precipitates, and the supernatant was collected. If the mice were found to be in poor activity and did not eat, they were immediately sacrificed for ascites. After collection and classification, they were stored in a -80°C refrigerator.

### 2.4. Purification of Ascites Antibodies

The antibody ascites fluid frozen at -80°C were thawed at 4°C overnight, centrifuged at 10,000 g at 4°C for 15 min, and removed the surface oil. The supernatant was passed through a membrane (0.22um) and stored at 4°C for later use and. Dilute with sufficient amount of Binding Buffer. The column and buffer were equilibrated to room temperature, centrifuged the stored antibody ascites fluid at 1000 g for 1 min, and removed the storage solution. A total of 2 mL of Binding Buffer was added to equilibrate the column, centrifuged for 1 min, discarded the liquid flowing through the column, and repeated once. The bottom of the column was covered with a rubber cap, the sample was put on the column, and its top was covered tightly. The column was mixed gently for 10 minutes at room temperature. The top cap was loosed gently, and the bottom cap was removed. The column was placed in a 15 mL collection tube and centrifuged for 1 min to collect the liquid. The column was then transferred to a new 15 mL centrifuge tube, and 2 mL of binding buffer was added, centrifuged for 1 min, and repeated the washing 3 times. Then, 100 *μ*l of neutralization buffer was added to three 15 mL collection tubes, respectively, and put the spin column into one of them. Elution buffer (1 mL) was added to the column and centrifuged for 1 min. The column was transferred to another collection tube containing neutralization buffer. The collected solution was saved as the first elution fraction and repeated this step 3 times to obtain 4 purified fractions. Fractions containing purified antibodies and content were determined by measuring the relative absorbance of each fraction at 280 nm [10, 11].

The article "Purification and Analysis of the CREPT Antibody from Mouse Ascites" was retracted in 2023. Reasons: signs of a paper mill; suspected computer-generated content; unreliable results or conclusions; concerns about the data.

### 2.5. SDS-PAGE Analysis

Protein concentration was determined according to the method of BCA protein concentration determination. Undenatured solution was taken at each stage of purification and used the BCA protein concentration determination kit to measure the protein concentration following the kit instructions. 10% separating gel and 5% stacking gel were put on the gel maker for use. The purified antibody protein was added to SDS-PAGE Sample Loading Buffer (5×) at a ratio of 4 : 1, followed by a boiling water bath for 10 min. According to the method of SDS-PAGE [12], the gel was put into the electrophoresis tank, and electrophoresis solution was added and loaded the sample for electrophoresis. The electrophoresis conditions were 80 V for stacking gel and 120 V for separating gel. Bromophenol blue was observed during electrophoresis, and electrophoresis was stopped when it was about 1 cm from the bottom. The gel was taken out, washed, fixed, stained with Coomassie brilliant blue, and destained, and the bands were observed and photographed.

### 2.6. Extraction of Total Protein from MOLT-4 Cells

MOLT-4 cell culture medium was composed of 10% FBS, 2% PS, and 88% 1640 basal medium. According to the culture method stated above, MOLT-4 was collected in the logarithmic growth phase and centrifuged at 3200 rpm for 5 min to discard the supernatant and collect the cell pellet. After counting, 250 *μ*L (10^6^ cells) of RIPA lysis solution was added, shaken, and put in ice bath for 30 minutes. During the ice bath, pipetting and mixing were repeated to completely lyse. Finally, they were centrifuged at 12,000 rpm and 4°C for 10 min and collected the supernatant as MOLT-4 cell total protein solution [13].

### 2.7. Identification and Analysis of Western Blot

The gel was prepared according to the method stated above for SDS analysis. The sample loaded was MOLT-4 cell total protein solution. After electrophoresis, transfer the membrane, immunoadsorption reaction (primary antibody: purified 3E10 CREPT monoclonal antibody protein was used in the test group, and RPRD1B antibody was used in the control group; secondary antibody: horseradish peroxidase-labeled goat anti-mouse IgG), and chemiluminescence (put the membrane into the developing apparatus, mixed the ECL solution A and B solution in equal volumes, and add sufficient ECL solution on the membrane to react for 2 min). The specific binding ability was detected by western blot in the GE multifunctional gel imager [14].

The article "Purification and Analysis of the CREPT Antibody from Mouse Ascites" was retracted in 2023. Reasons: signs of a paper mill; suspected computer-generated content; unreliable results or conclusions; concerns about the data.

## 3. Results

### 3.1. Monoclonal Cell 3E10 Cell Culture

Through cell activation culture, 10% FBS 1640 medium culture was added in a saturated humidity incubator at 37°C and 5% CO_2_ atmosphere. The culture medium was changed every 2-3 days, and the cells were observed. The monoclonal 3E10 cells in the logarithmic growth phase were obtained, which were plump, round, and smooth, and were semiadherent cells, as shown in Figure 1.

### 3.2. Preparation and Results of Mouse Ascites

Female mice were sensitized with incomplete Freund's adjuvant intraperitoneally for 7-15 days. The cells in the logarithmic growth phase were injected intraperitoneally with 1 mL/mouse at 10^6^ cells/mL, and flowable ascites appeared in the abdomen of the mice for about 7 days. Ascites were collected multiple times between 7 and15 days as shown in Figure 2(a), centrifuged to collect, and cryopreserved as shown in Figure 2(b).

### 3.3. Purification of Ascites Antibodies

The antibodies from ascites were purified through the collection, filtration, dilution, sample loading, and chromatography, and a 4-component antibody-protein solution was obtained. Purity and molecular weight were identified by SDS-PAGE. The maximum concentration of the purified antibody-protein sample was 1895 *μ*g/mL. As shown in Figure 3, lane 1 is the unpurified ascites sample, lane 2 is the unbound sample after loading, lane 3 is the maker, and lanes 4-7 are the eluted target proteins. The purified antibody has 2 bands, the possible reason is that one is a heavy chain with a size of about 37 kDa, and the other is a light chain. This is because the disulfide bonds between the immunoglobulin heavy and light chains are reduced by the action of mercaptoethanol. The size of the obtained antibody was consistent with the size of the target protein. It can be seen from the purification results that most of the impurity proteins are removed to obtain antibody proteins with higher purity and better activity. A one-step purification method for ascites monoclonal antibody was established to obtain CREPT ascites antibody with high activity and high purity.

### 3.4. Extraction of Total Protein from MOLT-4 Cells

Total protein from MOLT-4 cells was extracted using RIPA lysis buffer. The MOLT-4 cells were extracted in the logarithmic growth phase to obtain a total protein solution and then performed western blot analysis after protein concentration determination.

The article "Purification and Analysis of the CREPT Antibody from Mouse Ascites" was retracted in 2023. Reasons: signs of a paper mill; suspected computer-generated content; unreliable results or conclusions; concerns about the data.

### 3.5. Identification and Western Blot Analysis

Through the western blot analysis, the total protein of MOLT-4 cells was loaded as the sample (Figure 4), and the antibodies were primary antibody: the test group used purified 3E10 CREPT monoclonal antibody protein, and the control group used RPRD1B antibody: secondary antibody: horseradish peroxidase-labeled goat antibody mouse IgG. By chemiluminescence development, the results are shown in Figure 5. Figure 5(a) shows the purification component 1 of the experimental group. The primary antibody is diluted 1 : 200; Figure 5(b) shows the purification component 2 of the experimental group where the primary antibody was diluted 1 : 200. Figure 5(c) is the experimental group purification component 3 where the primary antibody was diluted 1 : 200. Figure 5(d) is for the experimental group purification component 4 where the primary antibody is diluted 1 : 200. Figure 5(e) is the control group, and the primary antibody was RPRD1B antibody and diluted 1 : 4000. From the results, it can be concluded that specific bands appeared in both the control group and the experimental group, indicating that the protein purified from ascites fluid is a CREPT monoclonal antibody protein, which is active and has high purity. It can specifically bind to the target protein in the western blot experiment, providing basic data for further research.

## 4. Discussion

With the increase in the incidence of cancer, the research on its pathogenesis has become more and more in-depth in recent years. The occurrence and development of tumors are closely related to the cell cycle. The CREPT gene, also known as RPRD1B, was discovered in 2010. After previous experimental verification, CREPT has been found in a variety of cancer tissues, such as lung cancer, gastric cancer, and colorectum. It is a protooncogene, which is highly expressed in cancer tissues and low in adjacent tissues [7].

CREPT, which is abundantly expressed through cell cycle regulation, accelerates the growth of tumor cells. However, the low expression of CREPT reduces tumor growth rate [15]. Mei Kunrong's ChIP experiment also showed that CREPT binds to the promoter of cyclin (cyclin D1) during the cell cycle and accelerates its transcription, thereby increasing the expression level of cyclin D1. In turn, it participates in the regulation of the cell cycle [16], increases the formation of clones, promotes the proliferation of cancer cells, and accelerates the G1/S transition of the cell cycle. In addition, 3C experiments demonstrated that CREPT regulates the transcription of cyclin D1 through the formation of chromatin loops [17, 18].

The article "Purification and Analysis of the CREPT Antibody from Mouse Ascites" was retracted in 2023. Reasons: signs of a paper mill; suspected computer-generated content; unreliable results or conclusions; concerns about the data.

In this study, by injecting monoclonal antibody cells into mice, a large number of antibodies were obtained and purified through the production of fluid ascites in the peritoneal cavity of mice. The purpose of this study was to obtain a highly purified antibody (purity of 1895 *μ*g/mL) and to perform a Western Blot validation study in lymphoma MOLT-4 cells with RPRD1B antibody as a control. The findings of this study are identical to those found in other oncology studies [19, 20]. Experiments also proved that CREPT is also expressed in lymphoma. CREPT may promote the proliferation of lymphoma cells and inhibit their differentiation by combining with related transcription factors, thereby promoting the occurrence of T-cell lymphoma. CREPT is highly expressed in T-cell lymphomas and can enhance the self-replication and metastasis abilities of lymphoma cells. The current research is still insufficient. In future, we aim to analyze the specific binding of CREPT to transcription factors and key target signaling pathways. In addition, we also aim to analyze the correlation between CREPT and the development of T-cell lymphoma, determine the relationship between high expression of CREPT and T-cell lymphoma, and provide a theoretical basis for CREPT as a potential drug target for the treatment of T-cell lymphoma. Purification of CREPT monoclonal antibody from ascites is for the first time to report from mouse ascites and obtain high-purity and high-activity antibody protein. The method is simple to prepare and provides a basis for further research on how CREPT affects the occurrence and development of tumors in the future.

## 5. Conclusion

This study was aimed at establishing a method for purifying CREPT from mouse ascites.

Cells were cultivated properly to obtain 3E10 crept monoclonal antibody cells in the logarithmic growth stage. Monoclonal antibody cells were injected into the abdominal cavity of sensitized mice. The flowing ascites were observed for 7-15 days. The antibody protein was obtained by collection, filtration, dilution, loading, and chromatography. Furthermore, its binding force was detected by SDS-PAGE and western blot techniques. The antibody protein was successfully obtained with a purity of 1895 *μ*g/mL with high liveness. This study establishes a one-step purification method for obtaining monoclonal antibody with high liveness and purity for CREPT ascites antibody. This method is simple to perform and lays a foundation for the preparation and purification of humanized monoclonal antibodies in the future. In addition, it provides a basis for further research to investigate how CREPT affects the occurrence and development of different tumors.

The article "Purification and Analysis of the CREPT Antibody from Mouse Ascites" was retracted in 2023. Reasons: signs of a paper mill; suspected computer-generated content; unreliable results or conclusions; concerns about the data.

## Figures and Tables

**Figure 1:** Cultured monoclonal antibody cell (3E10) observed under cell inverted microscope (IX73 + DP22 Olympus).

**Figure 2:** (a) Mouse ascites and (b) representation of the collected ascites.

**Figure 3:** Protein purification and SDS-PAGE analysis.

**Figure 4:** MOLT-4 cell culture (observed under cell inverted microscope (IX73 + DP22 Olympus).

**Figure 5:** Western blot results of the test and control groups.

## Data Availability

Data will be provided on request.
